# Synthesis, solvent role, absorption and emission studies of cytosine derivative

**DOI:** 10.1016/j.heliyon.2024.e28623

**Published:** 2024-03-26

**Authors:** N. Elangovan, Natarajan Arumugam, Abdulrahman I. Almansour, Shanty Mathew, Sinouvassane Djearamane, Ling Shing Wong, Saminathan Kayarohanam

**Affiliations:** a Research Centre for Computational and Theoretical Chemistry, Anjalam, 621208, Musiri, Tiruchirappalli, Tamilnadu, India; b Department of Chemistry, College of Science, King Saud University, P.O. Box 2455, Riyadh 11451, Saudi Arabia; c Department of Chemistry, St. Joseph's College Research Center, Shanthinagar, 560027, Bangalore, India; d Department of Allied Health Sciences, Faculty of Science, Universiti Tunku Abdul Rahman, Jalan Universiti, Bandar Barat, Kampar, 31900, Malaysia; e Biomedical Research Unit and Lab Animal Research Centre, Saveetha Dental College, Saveetha Institute of Medical and Technical Sciences, Saveetha University, Chennai, 602 105, India; f Faculty of Health and Life Sciences, INTI International University, Nilai, 71800, Malaysia; g Faculty of Bioeconomics and Health Sciences, University Geomatika Malaysia, Kuala Lumpur, 54200, Malaysia

**Keywords:** Synthesis, Cytosine, DFT, Molecular docking, Topology

## Abstract

The (E)-4-((4-hydroxy-3-methoxy-5-nitrobenzylidene) amino) pyrimidin-2(1H)-one (C5NV) was synthesized from cytosine and 5-nitrovanilline by simple straightforward condensation reaction. The structural characteristics of the compound was determined and optimized by WB97XD/cc-pVDZ basis set. The vibrational frequencies were computed and subsequently compared to the experimental frequencies. We investiated the electronic properties of the synthesized compound in gas and solvent phases using the time-dependent density functional theory (TD-DFT) approach, and compared them to experimental values. The fluorescence study showed three different wavelengths indicating the nature of the optical material properties. Frontier molecular orbital (FMO) and molecular electrostatic potential (MEP) analyses were conducted for the title compound, and electron localized functions (ELF) and localized orbital locators (LOL) were used to identify the orbital positions of localized and delocalized atoms. Non-covalent interactions (H-bond interactions) were investigated using reduced density gradients (RDGs). The objective of the study was to determine the physical, chemical, and biological properties of the C5NV. The molecular docking study was conducted between C5NV and 2XNF protein, its lowest binding energy score is −7.92 kcal/mol.

## Highlights

• Structural determination of novel compound (C5NV) was derived from cytosine.
• Electronic properties of C5NV compound was investigated by TD-DFT in gas and solvent phases.
• The active sites and interaction were determined by MEP, ELF, LOL, and RDG.
• The C5NV shows a good fluorescence spectrum indicating it is an optical material.
• FMO and MEP analysis were performed under various solvent system.

## 1 Introduction

Cytosine is one of the nucleobases found in DNA and RNA (or uracil in the case of RNA), and is categorized alongside adenine, guanine, and thymine. Watson-Crick base pairing involves the nucleotide adenine forming three hydrogen bonds with the nucleotide guanine [1]. The discovery and nomenclature of cytosine can be attributed to Albrecht Kossel and Albert Neumann in 1894, following its hydrolysis from tissues of the calf thymus. In the year 1903, a postulated structure was subsequently synthesized and the structure was then confirmed in the laboratory. A quantum information processing experiment from Oxford University was performed in 1998. The synthesis of cytosine, uracil, and thymine was discovered by NASA scientists in March 2015. These nucleobases were shown to be produced from pyrimidine under laboratory circumstances that mimic the environment of outer space [2]. A significant aspect of this discovery is the presence of pyrimidine in meteorites, despite uncertainty surrounding its origin.

Cytosine is present within DNA, RNA, and nucleotides. In its capacity as cytidine triphosphate (CTP), it exhibits co-factor activity with enzymes, facilitating the transfer of a phosphate group to convert ADP into ATP [3]. Cytosine forms a base pair with guanine in both DNA and RNA molecules. Nevertheless, it possesses inherent instability, rendering it susceptible to spontaneous deamination, resulting in the conversion to uracil [4]. If left unaddressed, this circumstance has the potential to result in a point mutation, until rectified by DNA repair enzymes like uracil glycosylase, which is responsible for the cleavage of uracil inside DNA. Cytosine can undergo methylation, resulting in the formation of 5-methylcytosine, a process facilitated by the enzyme DNA methyltransferase [5]. Additionally, cytosine can undergo both methylation and hydroxylation, leading to the production of 5-hydroxymethylcytosine [6]. Bisulfited sequencing is predicated upon the disparity in deamination rates between cytosine and 5-methylcytosine, leading to the conversion of the former to uracil and the latter to thymine [7].

Recently, synthesis, computational investigation and docking simulation of new class of Schiff base, 4,5-difluoro-2-((*m*-tolylimino)methyl)phenol was reported by Songul Sahin [8]. The mesomorphic properties of Schiff base, 6-aminocoumarin derivatives synthesized and characterized using POM and DSC analysis have been reported by Jayashree et al. [9]. A recent study by Marwa Benmabrouk et al. reported the structural determination, characterization, and antioxidant potential of Salicylideneaniline Schiff base [10]. Mira Patel et al. reported the discovery of a new class of curcumin Schiff bases as potential antibacterial agents [11].

A literature review shows that the C5NV compound has no reported physical, chemical, computational, biological properties. Hence, the present study synthesized and characterized the physical, chemical, and biological properties of C5NV compound in both experimental and theoretical methods.

## 2 Experimental

### 2.1 Materials and methods

The product referred to as C5NV was acquired from Sigma-Aldrich, a chemical corporation based in the United States. The compound obtained was of 99% purity and was utilized in its original state to record FT-IR and UV–visible spectra. The IFS 66V spectrophotometer is employed in this study, utilizing the K–Br (potassium bromide) pellet technique for solid phase analysis. The instrument was operated at a resolution of 4.0 cm^−1^ in evacuation mode, allowing for the recording of IR spectra within the range of 4000-400 cm^−1^. The absorption spectra of the sample were recorded using the JASCO V-670 Spectrometer, which operates in the wavelength range of 200–800 nm. The NMR was recorded from Bruker advanced 400 MHz.

### 2.2 Synthesis of (E)-4-((4-hydroxy-3-methoxy-5-nitrobenzylidene) amino) pyrimidin-2(1H)-one (C5NV)

By using the mechanic-grinding method, the Schiff base (E)-4-((4-hydroxy-3-methoxy-5-nitrobenzylidene) amino) pyrimidin-2(1H)-one (C5NV) had to be made by cytosine and 5-nitrovanilline. About 1:1 mol ration of cytosine and 5-nitrovanilline were added. It was mixed with one drop of acetic acid, and after some more grinding, a yellow solid was found. Using ethanol as a solvent, the powder was put into a beaker and heated in a water bath until the mixture was uniform. The solvent was then let to evaporate by leaving the mixture alone for a while. The finished item was then cleaned, filtered, and made crystal clear using DMSO [8,9]. Scheme 1 is illustrated within the reaction procedure.

**Scheme 1:** Synthesis of (E)-4-((4-hydroxy-3-methoxy-5-nitrobenzylidene) amino) pyrimidin-2(1H)-one (C5NV).

### 2.3 Molecular docking protocol

The docking process utilized the Lamarckian genetic algorithm (LGA) to establish the docking configuration. The resulting conformations were evaluated and grouped based on their similarities in conformation and root-mean-square positional deviation (RMSD). The run count was standardized to 10 for the titled compound. The root mean square deviation (RMSD) was computed using a conformational clustering tolerance of 2.0 Å. The settings for the genetic algorithms were configured as follows: a population size of 150, a mutation rate of 0.02, a crossover rate of 0.8, a maximum number of generations of 27000, and a maximum number of energy evaluations of 2500000. The LGA docking process utilized the pseudo-Solis and Wets local search method, with a maximum of 300 iterations per local search. The probability of performing a local search on an individual in the population was set to 0.06. The maximum number of consecutive successes or failures before doubling or halving the ρ was four for both. Lastly, the lower bound on ρ was set to 0.01.

### 2.4 Computational methods

The Gaussian software was employed to conduct the theoretical calculations [10]. A standard cc-pVDZ basis set was employed [11]. Density functional theory (DFT) was implemented specifically WB97XD theory. Consequently, the frequencies and infrared intensity are determined without scaling [12]. To align the theoretical frequencies with the experimental frequencies, a scaling factor of 0.9651 cm^−1^ is applied to the vibrational frequencies [13]. Once the scaling factor is applied, the departure from the experimental results becomes more dependable. The vibrational assignments have been conducted using the same theoretical framework [14]. The VEDA 4.0 program package was utilized to do the computation of potential energy distribution (PED) and the determination of vibrational frequency assignments. The software Multiwfn was used to calculate the ELF, LOL, and RDG studies [15]. Using autodock-4 software the titled compound molecular docking was conducted.

## 3 Results and discussion

### 3.1 Structural geometry analysis

The present study focuses on the optimization of the C5NV molecule by the DFT method. Specifically, the dispersion correction method WB97XD was employed, to carry out the optimization process [16]. The presence of an imaginary frequency in the molecular system indicates the lack of negative frequencies, so confirming that the system has undergone complete optimization and convergence [17]. Fig. 1 illustrates the structure of C5NV, with the atoms appropriately numbered [18]. Table S1 presents the geometrical parameters of the titled compound [19]. It is observed that the optimized structure associated with the lowest energy E = −1058.043836 a.u) is produced using the WB97XD/cc-pVDZ technique [20]. The molecule being examined demonstrates an overall arrangement of seven C–H bond lengths, two O–N bond lengths, one N–H bond length, nine C–C bond lengths, and four O–C bond lengths [21]. There is a total of nine carbon-carbon (C–C) bond lengths within the phenyl ring. In the context of DFT, these bond lengths range from 1.3582 to 1.4628 A°. The bond length of C3–C7 (1.4628 A°) exhibits greater magnitudes than the remaining C–C bond lengths inside the ring [22]. The lengths of C–H bonds exhibit elongation within the range of 1.0894–1.1023 A° as determined by DFT [23]. The bond lengths N19–O21 and N19–O20, as determined by DFT calculations, are determined to be 1.2188 A° and 1.2132 A°, respectively.

**Fig. 1:** Optimized structure of C5NV.

### 3.2 Vibrational analysis

The vibrational spectra simulations of the C5NV molecule were conducted by employing the optimized geometry of C1 through density functional theory (DFT) calculations [24,25]. Table 1 presents a comparison between the theoretical IR bands obtained at the WB97XD/cc-pVDZ level and the experimental FTIR bands for several significant theoretical IR bands [26]. In general, it is seen that the harmonic frequencies tend to exceed the experimental frequencies [27]. There is a consistent occurrence of overestimation observed in the comparison of theoretical and experimental IR frequencies [28]. Consequently, researchers have utilized several scaling procedures to align the theoretical position of the IR band with the corresponding experimental data [29]. In the present study, a uniform scaling factor of 0.9651 was employed to reduce the magnitude of the harmonic wavenumbers [30]. The generated infrared spectra have been compared to the experimental spectrum, as depicted in Fig. 2.

**Table 1:** Experimental and theoretical FTIR wavenumbers and PED analysis of C5NV.

WB97XD/cc-pVDZ					Observed	Assignment (% PED)
Mode	Unscaled	Scaled	IRI	RA	IR	
87	3759.8	3628.583	200.99	130.59	3589	νNH(100)
86	3653.24	3525.742	129.66	169.87	3354	νOH(99)
85	3279.03	3164.592	1.3029	84.588	3194	νCH(98)
84	3249	3135.61	5.5604	20.97	–	νCH(99)
83	3247.15	3133.824	7.3417	42.094	–	νCH(99)
82	3233.65	3120.796	3.6716	146.55	3095	νCH(98)
81	3186.81	3075.59	12.966	133.5	3080	νCH(89)
80	3120.42	3011.517	22.774	38.433	3030	νCH(100)
79	3099.37	2991.202	5.9659	28.5	2985	νCH(100)
78	3035.31	2929.378	35.076	123.47	2924	νCH(89)
77	1857.18	1792.364	737.77	20.045	1734	νOC(76)
76	1742.98	1682.15	36.749	649.98	1681	νNC(16)+νCC(33)
75	1731.84	1671.399	249.42	467.23	1665	νCC(46)
74	1696.68	1637.466	903.7	350.01	–	νCC(50)+βHOC(10)
73	1690.85	1631.839	253.81	987.06	–	νNC(52)+βHCN(10)
72	1676.44	1617.932	98.867	575.59	1603	βHCH(72) + HCOC(22)
71	1613.68	1557.363	220.45	136.99	1577	βHCH(75) + HCOC(17)
70	1573.62	1518.701	244.42	35.173	1548	νCC(39)+βHNC(14)
69	1515.23	1462.348	33.882	38.878	1460	νCC(15)+νOC+10)+βHCH(33)
68	1507.37	1454.763	199.43	535.27	–	βHCH(42)
67	1486.92	1435.026	111.97	15.031	–	νCC(11)+βHCH(11)
66	1480.91	1429.226	250.78	23.849	–	νCC(17)+βHCC(19)+βHCN(18)
65	1473.45	1422.027	9.8884	17.564	–	βHOC(26)
64	1464.21	1413.109	76.251	59.019	1413	νCC(19)+βHNC(42)
63	1456.34	1405.514	79.751	44.351	1401	βHCN(48)
62	1438.78	1388.567	176.63	104.62	1383	νON(77)
61	1383.91	1335.612	124.98	0.4642	1360	νCC(19)+βHOC(20)+βHCC(13)
60	1342.78	1295.917	147.41	52.24	–	νCC(37)+βHCN(10)
59	1329.25	1282.859	177.1	26.909	1268	νNC(44)
58	1305.09	1259.542	28.76	30.872	–	νCC(15)+βHCN(36)
57	1295.05	1249.853	251.99	399.75	1234	νNC(15)+νOC(11)+βHCC(15)
56	1238.04	1194.832	27.393	41.638	1199	νCC(12)+βHNC(13)
55	1229.37	1186.465	27.216	77.843	1190	βHCH(20)+τHCOC(63)
54	1210.6	1168.35	141.56	35.099	–	νON(51)+βCCC(10)
53	1205.44	1163.37	98.002	14.274	1163	βHCH(25)+τHCOC(38)
52	1178.52	1137.39	145.7	70.439	1134	νCC(10)+νOC(11)+βHNC(16)
51	1173.83	1132.863	0.7055	1.6469	1104	νNC(50)+βHCC(11)
50	1117.36	1078.364	6.1431	6.8874	–	νCC(50)+βHCC(22)
49	1114.97	1076.058	57.212	44.062	–	τHCNC(81)
48	1054.05	1017.264	12.018	2.8065	1049	νOC(38)+βCCC(10)
47	1029.66	993.7249	27.789	40.102	–	τHCCN(71)
46	1022.46	986.7761	4.3109	6.9362	973	τHCCC(72)
45	986.54	952.1098	0.1187	1.2065	953	τHCCC(76)
44	972.53	938.5887	0.0789	59.182	–	νOC(58)
43	957.19	923.7841	90.085	20.639	918	νNC(24)+βCCC(32)
42	939.02	906.2482	1.2998	2.4142	–	βCCN(45)
41	922.56	890.3627	22.853	2.995	896	νNC(49)
40	850.9	821.2036	4.4847	8.3532	–	τHCCN(58)+τHNCN(22)+τCCCN(10)
39	833.36	804.2757	47.374	17.873	–	τNCCC(68)
38	813.95	785.5431	41.939	7.244	–	τCCCN(70)
37	804.95	776.8572	4.5239	3.3056	874	νOC(17)+βCCC(20)
36	795.8	768.0266	18.649	2.6145	–	νNC(10)+νCC(10)+βCCC(10)+βCCN(10)
35	786.08	758.6458	14.023	2.3491	–	τHCCN(20)+τHNCN(57)
34	755.8	729.4226	34.941	4.6432	–	νON(10)+βCCC(47)
33	740.35	714.5118	1.3849	0.9442	–	τHNCN(70)
32	697.25	672.916	27.339	3.5142	–	τHNCN(77)
31	674.29	650.7573	32.18	2.8712	–	βCCN(22)
30	659.85	636.8212	7.6325	4.2079	–	τHOCC(90)
29	629.65	607.6752	27.285	0.2705	–	βCCC(38)+τCCCC(19)
28	586.67	566.1952	1.9	3.6268	–	τCCCC(11)
27	574.66	554.6044	21.587	2.6826	–	βCNC(64)
26	571.11	551.1783	80.274	2.5277	–	νCC(22)+βCCC(17)
25	563.56	543.8918	4.1502	2.7402	–	βCCC(10)+βCNC(37)
24	522.39	504.1586	3.4391	0.9003	–	τCCCC(67)
23	516.39	498.368	3.7332	1.2934	–	νOC(13)+βCCN(24)+βCCC(12)
22	464.09	447.8933	2.4455	0.3886	–	τHCCN(11)+τCCCN(55)
21	441.02	425.6284	3.4781	3.6699	–	βCNC(47)
20	428.23	413.2848	8.7625	8.4489	–	τCCCC(11)+τCCCN(51)
19	407.75	393.5195	1.2856	5.9127	–	βONC(44)
18	383.7	370.3089	1.3301	3.7997	–	βCCC(14)+βCCO(14)+βONC(14)
17	360.84	348.2467	8.5536	8.7957	–	βCCO(38)+βCCC(12)
16	312.04	301.1498	5.4935	2.0559	–	τCCCC(48)
15	285.14	275.1886	0.6534	0.7652	–	βCCC(28)+βONC(12)
14	260.3	251.2155	0.236	6.9351	–	τCCCC(23)
13	237.88	229.578	3.6352	7.619	–	τCCCN(62)
12	228.31	220.342	3.5469	0.5504	–	βCCN(32)
11	206.51	199.3028	0.3419	2.9772	–	τHCOC(41)+τCCCC(15)
10	178.52	172.2897	3.9859	0.4395	–	βCCN(53)
9	145.58	140.4993	0.6293	5.3033	–	τCCCN(75)
8	133.91	129.2365	6.0118	1.8438	–	βCCC(12)+βCOC(61)
7	123.88	119.5566	6.4993	1.098	–	τCCCC(34)+τCCNC(14)
6	103.16	99.55972	7.0537	4.8938	–	τCCCN(12)+τCCCC(12)+τCCNC(11)
5	65.33	63.04998	1.4312	0.0729	–	τCCNC(64)+τCCCC(10)
4	47.63	45.96771	0.6009	2.1541	–	τCCCC(69)+τCCNC(12)
3	44.11	42.57056	0.991	0.4777	–	βCCC(86)
2	28.9	27.89139	0.1792	1.8066	–	τCCCC(68)
1	21.77	21.01023	3.4487	3.8375	–	τCCNC(77)

**Fig. 2:** Comparison (experimental and theoretical) FTIR spectrum of C5NV.

### 3.3 N–H vibration

The absorption of primary amine occurs within the spectral range of 3500-3300 cm^−1^, in the N–H bond. The νNH stretching vibration is detected at 3589 cm^−1^ in the experimental FTIR [31]. The scaled wavenumber has appeared in 3628 cm^−1^ and the %PED is 100%. The experimental βHCN bending vibrations are 1548, 1413, 1401, 1199, and 1134 cm^−1^, and calculated bending vibrations are 1637, 1518, 1429, 1413, 1405, 1295, 1259, 1194, and 1137, %PED are 10, 14, 18, 42, 48, 10, 36, 13 and 16 respectively. The calculated torsion vibrations (τHCCN) are 993, 821, and 758 cm^−1,^ and % PEDs are 71, 58, and 20 respectively.

### 3.4 C–H vibration

Typically, infrared bands exhibiting moderate to high intensity as a result of alkene CH stretching vibrations are observed within the spectral range of 3100-3000 cm^−1^ [32]. The experimental CH vibrations are 3194, 3095, and 3030 cm^−1^ and the calculated CH stretching vibrations are 3164, 3135, 3133, 3120, 3075, and 3011 cm^−1^ and %PEDs are 98, 99, 99, 95, 100, 100, and 89 respectively. The alkane CH stretching vibrations range from 3000 cm to 1 to 2840 cm-1. The experimental CH vibrations are 2985 cm^−1^ and 2924 cm^−1^, and the calculated vibrations are 2991 cm^−1^ and 2929 cm^−1^, with %PED is 100 and 89 respectively. The experimentally observed bending vibrations are 1603, 1557, 1460, and 1190 cm^−1,^ and calculated bending vibrations are 1617, 1557, 1462, 1454, 1435, and 1186 cm^−1^, with %PED 72, 75, 33, 42, 11 and 20 respectively. The experimental torsion vibrations are 1603, 1577, and 1163 cm^−1^ and the calculated are 1617, 1557, 1163, and 199 cm^−1^, with %PED 42, 17, 38, and 41 respectively.

### 3.5 C–C vibration

The C–C stretching vibrations are experimentally observed in the range of 1665, 1540, 1460, and 1360 cm^−1^ and the calculated stretching vibrations are 1671, 1637, 1518, 1462, 1432, 1429, 1413, 1335, 1295, 1259, 1194, 1137 and 1078 cm^−1^, with %PED 46, 50, 95, 15, 11, 17, 19, 19, 37, 15, 12, 10, 50 and 22 respectively. The calculated bending and torsion vibrations are 1168, 1017, 923, 776, 768, 729, 607, 551, 543, 498, 370, 75, 129, 42 cm^−1^, and 607, 566, 504, 413, 301, 251, 199, 119, 99, 63, 45, 27 cm^−1^, with %PED 10, 10, 32, 20, 10, 47, 38, 17, 10, 12, 14, 28, 12, 86 and 19, 11, 67, 11, 48, 23, 15, 34, 12, 10, 69, 68 respectively.

### 3.6 O–H vibration

The calculated OH stretching vibration is 3525 cm^−1^, whereas the experimentally observed OH stretching vibration is 3354 cm^−1^; the PED contribution is 99%. The experimental and theoretical bending vibrations are 1335 cm^−1^ and 1360 cm^−1^, respectively, with a PED of 20%. Experimentally observed torsion vibrations are 973 cm^−1^ and 953 cm^−1^, whereas their theoretical values are 986 cm^−1^ and 952 cm^−1^, with respective PED values of 72% and 76% respectively.

### 3.7 N–C vibration

The NC stretching vibrations experimentally observed are 1681, 1268, 1234 1104, and 896 cm^−1^, and calculated vibrations are 1682, 1631, 1282, 1249, 1132, 890, and 768 cm^−1^, with %PED 16, 52, 44, 15, 50, 49 and 10 respectively [33]. The calculated CCN bending vibrations and CCCN torsion vibrations are 906, 768, 650, 544, 543, 498, 425, 220 and 172 cm^−1^, and 821, 447, 413, 229, 119, 97, 45, 21 cm^−1^ with % PED 45, 10, 22, 64, 37, 24, 47, 32 and 53, and 10, 68, 55, 51, 62, 14, 11, 12, 77 respectively.

### 3.8 O–N and O–C vibration

The ON experimental starching vibration is 1383 cm^−1^ and the calculated NO stretching vibrations are 1388, 1168, and 729 cm^−1^, with % PED, 77, 51, and 10 respectively [34]. The calculated bending torsion vibrations are 968, 650, 554, 543, 498, 425, 220, 172 cm^−1^, and 821, 804, 447, 413, 29, 119, 97, 45, 21 cm^−1^, with %PED 45, 10, 22, 64, 37, 24, 47, 32, 53, and 10, 68, 55, 51, 62, 14, 11, 12, 77 respectively. The experimental CO stretching vibrations are 1734, 1134, 1049, and 874 cm^−1^ and calculated values are 1792, 1137, 1017, 938, 776, and 498 cm^−1^, with % PED, 76, 11, 38, 58, 17, and 13. The calculated bending vibration is 1637 cm^−1^, with a % PED is 10.

### 3.9 NMR spectral analysis

NMR spectroscopy is an influential analytical technique employed for the examination of molecular structure and dynamics. NMR spectra yield data regarding the nuclear surroundings of certain atoms within a given sample [35]. Chemical shift is a measure of the electronic surroundings of a nucleus [36]. Protons that have been deshielded due to electron-withdrawing environments are observed at lower chemical shifts, whereas shielded protons in electron-donating settings are observed at higher chemical shifts [37]. The quantity of peaks in a signal is directly linked to the quantity of adjacent, distinct protons that are not equivalent (N+1 rule). Examine the splitting pattern to ascertain the number of neighboring protons. A singlet, characterized by a single peak, indicates the absence of nearby protons. Conversely, a triplet, which exhibits three peaks, suggests the presence of two adjacent protons [38]. The occurrence of multiple patterns is a result of the interaction between neighboring nuclei through spin-spin coupling. For instance, a triplet may signify the connection to two identical protons. Verify that the integration values correspond to the anticipated ratio determined by the molecular formula [39]. The NMR is a very important one for an organic compound, in this study the theoretical section we used WB97XD/cc-pVDZ methods. The titled compound NMR spectral is presented in Fig. 3. The ^1^HNMR experimental observed chemical shifts are H25 is 9.73 ppm, H24 and H26 is 9.06 ppm, H22, and H23 is both 8.05 ppm, H27 and H28 are 7.69 ppm, and H29, H30, and H31 are 3.85 ppm. The calculated chemical shifts are 9.41, 8.64, 8.44, 8.04, 7.69, 7.03, 6.58, 4.67, 4.23 and 4.20 ppm respectively.

**Fig. 3:** ^1^HNMR spectra of C5NV.

### 3.10 Absorption (UV) spectral analysis

The C5NV was subjected to TD-DFT computations in the various phases using the WB97XD-cc-pVDZ method [40]. Table 2 presents the electronic absorption wavelengths, oscillator strengths, and excitation energy transitions of the aforementioned compound in the gas phase and diverse solvent phase [41]. A comparison UV visible study of C5NV with various solvents and gas phase is presented in Fig. 4. The compound C5NV exhibited an absorption band at a gas phase wavelength of 308, 293and 290 nm, and other solvents of chloroform, DMSO and water are absorption wavelengths of 305, 301, and 291 nm; 309, 299, and 292; and 308, 299 and 291 nm, respectively [42]. The titled compound showed two different wavelengths in the experimental section such as 256 nm and 274 nm respectively [43]. The absorption band observed at the gas phase wavelength of 308 nm exhibits an energy of 32718.68697 and oscillator strength of 0.2332, and the HOMO-LUMO contribution is H-6- > L+1 (57%), H-5- > L+1 (11%) H-6- > LUMO (6%), H-6- > L+3 (7%), H-3- > L+1 (9%), at 293 nm exhibits the energy of 34029.3379139 and oscillator strength of 0.3112, which is HOMO- > LUMO (50%), HOMO- > L+1 (18%) H-5 >LUMO (5%), H-2- > LUMO (6%), H-1- > LUMO (6%), H-1- > L+1 (4%), H-1- > L+2 (2%) and at a wavelength of 290 nm exhibits the energy of 34410.8381589 and oscillator strength of 0.0178, which contribution is H-5- > LUMO (10%), H-2- > LUMO (25%), H-1- > LUMO (19%), HOMO- > L+1 (12%) H-4- > LUMO (4%), H-3- > LUMO (4%), H-2- > L+1 (4%), H-2- > L+2 (2%), HOMO- > LUMO (7%). Table 2 has a listing of the HOMO and LUMO contributions made by these additional solvents, which include chloroform, DMSO, and water.

**Table 2:** UV visible absorption study and HOMO-LUMO contribution of C5NV with different solvents.

Media	Wavelength (nm)	Band Gap eV	Energy (cm-1)	Oscillator Strength	Contribution
Chloroform	305.6357369	2.73	32718.68697	0.2332	HOMO- > LUMO (57%), HOMO- > L+1 (24%)H-6- > L+1 (5%), H-1- > L+1 (3%)
	301.6867241		33146.96737	0.0599	H-6- > LUMO (12%), H-6- > L+1 (59%) H-6- > L+3 (6%), H-2- > L+1 (4%), HOMO- > LUMO (6%)
	291.5011709		34305.17953	0.3583	H-3- > LUMO (10%), H-1- > LUMO (33%), HOMO- > L+1 (25%) H-5- > LUMO (5%), H-4- > LUMO (2%), H-3- > L+1 (2%), H-1- > L+1 (5%), H-1- > L+2 (6%), HOMO- > LUMO (7%)
DMSO	309.1566752	2.73	32346.05882	0.1979	HOMO- > LUMO (63%), HOMO- > L+1 (24%) H-1- > L+1 (3%)
	299.5438453		33384.09437	0.033	H-6- > LUMO (19%), H-6- > L+1 (56%) H-7- > L+1 (3%), H-6- > L+3 (5%), H-2- > L+1 (4%)
	292.2914636		34212.42577	0.4805	H-1- > LUMO (26%), HOMO- > LUMO (10%), HOMO- > L+1 (30%) H-5- > LUMO (3%), H-4- > LUMO (3%), H-3- > LUMO (6%), H-3- > L+1 (2%), H-1- > L+1 (6%), H-1- > L+2 (6%)
Gas Phase	308.3263529	2.73	32433.1667	0.0031	H-6- > L+1 (57%), H-5- > L+1 (11%) H-6- > LUMO (6%), H-6- > L+3 (7%), H-3- > L+1 (9%)
	293.8640777		34029.33791	0.3112	HOMO- > LUMO (50%), HOMO- > L+1 (18%) H-5- > LUMO (5%), H-2- > LUMO (6%), H-1- > LUMO (6%), H-1- > L+1 (4%), H-1- > L+2 (2%)
	290.6061153		34410.83816	0.0178	H-5- > LUMO (10%), H-2- > LUMO (25%), H-1- > LUMO (19%), HOMO- > L+1 (12%) H-4- > LUMO (4%), H-3- > LUMO (4%), H-2- > L+1 (4%), H-2- > L+2 (2%), HOMO- > LUMO (7%)
Warer	308.9255818	2.73	32370.25545	0.1819	HOMO- > LUMO (62%), HOMO- > L+1 (25%) H-1- > L+1 (3%)
	299.3702596		33403.45168	0.0287	H-6- > LUMO (20%), H-6- > L+1 (56%) H-7- > L+1 (4%), H-6- > L+3 (5%), H-2- > L+1 (4%)
	291.7755701		34272.91735	0.4682	H-1- > LUMO (26%), HOMO- > LUMO (11%), HOMO- > L+1 (29%) H-5- > LUMO (3%), H-4- > LUMO (3%), H-3- > LUMO (6%), H-3- > L+1 (2%), H-1- > L+1 (7%), H-1- > L+2 (6%)

**Fig. 4:** UV visible spectrum of C5NV (a) chloroform, (b) DMSO, (c) Water and (d) experimental with chloroform.

### 3.11 Fluorescence spectroscopy

The phenomenon of fluorescence occurs when a substance absorbs light of a particular wavelength and subsequently releases light of an extended wavelength [44]. This process is commonly defined by the absorption of light with shorter wavelengths (more energy) and the emission of light with longer wavelengths (lower energy). The light that is released is frequently of a distinct hue from the light that is taken in Ref. [45]. Fluorescence commences when a substance absorbs photons, which are particles of light. The absorption of energy elevates the energy level of electrons within the atoms or molecules of the substance to a state of excitement [46]. The excited state is inherently unstable, prompting the electrons to go back to their lower energy state by the emission of light energy. The term used to describe this emitted light is fluorescence [47]. The light that is released usually has a greater wavelength than the light that is taken in. Fluorescence is extensively utilized in several disciplines such as biology, chemistry, medicine, and materials research. Fluorescent dyes are frequently employed to mark and observe particular molecules or structures in biological materials [48]. Fig. 5 shows the fluorescence spectrum of C5NV. Fluorescence is also employed in several industrial applications, including quality control and monitoring operations. Fluorescent markers and dyes are frequently employed in these applications to identify and examine particular compounds. This compound showed three different wavelengths such as 374 nm, 646 nm, and 727 nm respectively.

**Fig. 5:** Fluorescence spectra of C5NV.

### 3.12 Nonlinear optical properties (NLO)

Molecular-based materials exhibiting second-order nonlinear optical (NLO) properties have gathered important consideration in topical periods outstanding to their involvement in novel scientific phenomena and their prospective applications in growing fields such as optoelectronic technologies, telecommunications, optical switching, and signal processing [49]. The total dipole moment was determined using the implementation of DFT with the WB97XD functional and the cc-pVDZ basis set. It is noteworthy that the values of the title molecule are 3.72 times greater than those of urea [50]. Specifically, the titled compound values are measured using the WB97XD/cc-pVDZ method. Furthermore, the chloroform, DMSO, gas phase, and water dipole moments are 12.11, 12.90, 12.86, and 12.90, respectively. Based on this record the chloroform dipole moment is highest [51].

### 3.13 HOMO-LUMO analysis

The optical and electrical characteristics of the titled compound were obtained from utilization for FMO theory [52]. This theoretical framework also elucidates the diverse array of reactions that can occur inside conjugated systems [53]. The HOMO signifies the electron-donating ability, while the LUMO signifies the electron-accepting tendency, specifically in the context of nucleophilic behavior [54]. Fig. 6 depicts the molecular surfaces of the HOMO and the LUMO [55]. The gas phase LUMO is found to be predominantly localized within the titled compound, with a predicted energy of −0.22 eV. On the other hand, the HOMO is primarily localized within the titled compound, with a HOMO value of −0.32 eV. The energy gap of the gas phase, chloroform, DMSO, and water between the HOMO and the LUMO was calculated to be 2.73 eV [56]. The presence of a significant energy gap indicates that the crystal that has been cultivated possesses a high degree of stability, exhibits reduced chemical reactivity, and demonstrates diminished polarisation [57]. The remaining parameters were calculated and are presented in Table 3. The ionization potential is positively correlated with the energy value of the HOMO, while the electron affinity is positively correlated with the energy values of the LUMO [58]. An element with a greater ionization potential and electron affinity is indicative of a higher electronegativity value for that element [59]. Typically, the electron affinity is shown to be lower than the ionization potential, indicating a molecule's pronounced propensity for electron acquisition [60]. The quantification of a molecule's capacity to accept electrons is evaluated by the global electrophilicity index, which relies on the concepts of chemical potential and chemical hardness [61]. The observed low electrophilicity value of 6.01 eV further reinforces the notion of the produced material's strong stability and bioactivity, as previously reported [62]. The determination of the stability index of the compounds was accomplished through the assessment of the HOMO-LUMO energy gap, which concurrently offers insights into the wavelength at which the molecule is capable of absorbing.

**Fig. 6:** HOMO-LUMO (FMO) surface map of C5NV.

**Table 3:** Frontier molecular orbital (FMO) properties of C5NV.

Property	Gas Phase	Chloroform	DMSO	Water
ԑHOMO	−8.65	−8.65	−8.65	−8.65
ԑLUMO	−5.92	−5.92	−5.92	−5.92
ΔE	2.73	2.73	2.73	2.73
*I* = ԑHOMO = -HOMO	8.65	8.65	8.65	8.65
*A* = ԑLUMO = -LUMO	5.92	5.92	5.92	5.92
Ƞ = (*I-A*)/2	1.36	1.36	1.36	1.36
*S =1/Ƞ*	0.73	0.73	0.73	0.73
μ = -(I + *A*)/2	−7.28	−7.28	−7.28	−7.28
χ = -μ	7.28	7.28	7.28	7.28
ω = μ2/2Ƞ	6.01	6.01	6.01	6.01
*N* = 1/ω	0.16	0.16	0.16	0.16
ω+ = *A*2/2(*I-A*)	1.08	1.08	1.08	1.08
ω+ = *I*2/2(*I-A*)	1.58	1.58	1.58	1.58

### 3.14 MEP analysis

The MEP parameter is highly valuable in the identification of locations where electrophilic and nucleophilic reactions are likely to take place [63]. This parameter is closely linked to electronic density and the interactions that occur within a molecule. A color system was employed to distinguish between regions characterized by maximum negative potential, maximum positive potential, and intermediate potential zones [64]. The red color represents a negative, indicating a surface that is susceptible to electrophilic assaults. Conversely, the blue color represents a positive, indicating a surface that is conducive to nucleophilic attacks [65]. The various zones delineated by negative and positive potentials are visually distinguished through the utilization of distinct hues, such as yellow, green, and orange [66]. There is a possibility of observing incremental increases in the arrangement of colors, specifically in the order of red, orange, yellow, green, and blue [67]. The gas phase, chloroform, DMSO, and water MEP surfaces map are present in Fig. 7. This observation aligns with the anticipated propensity of this area to undergo electrophilic assaults.

**Fig. 7:** MEP surface map of C5NV.

### 3.15 NPA and MPA analysis

It is essential for understanding the charge distribution of a molecule to properly understand its electrostatic interaction, chemical reactivity, and molecular potential [68]. The MPA and NPA charges were employed methods for representing the electron distribution among atoms within a molecule [69]. These compounds identify atoms that receive electrons and become negative and atoms that lose electrons and become positive [70]. In addition, we conducted MPA and NPA to investigate the electrostatic potential and determine the electrophilic/nucleophilic characteristics [71]. Both the MPA and NPA techniques yielded comparable outcomes [72]. As anticipated, the predominant negative charges were primarily located on the nitrogen (N), and oxygen (O) atoms. Table 4 presents the MPA analysis of the titled compound and Table 5 presents the NPA analysis [73]. Fig. 8, Fig. 9 presents the graphical representation of C5NV. Hydrogen atoms and carbon atoms at positions C3, C6, C8, C9, and C10 exhibit significant positive charges. In NPA analysis all hydrogen atoms have positive charges. Generally, the highest positive charged and highest negative charged atoms are 0.87323 (C14) and −0.64674 (O8). This polarisation of bond charges can potentially contribute to the partial weakening of the bonds [74]. Atoms with the highest positive and negative charges exhibit pronounced regions of electrophilic and nucleophilic character within their structure, as well as the specific locations where hydrogen bond interactions occur [75]. All carbon atoms have positive charges except C3 and C14 in MPA analysis and the highest positive charge and the highest negative charge atoms are C14 (0.227604) and O17 (−0.346139). Also, all hydrogen atoms are positively charged.

**Table 4:** Mulliken population analysis (MPA) of C5NV.

Atom	Charge	Atom	Charge	Atom	Charge	Atom	Charge
1 C	0.107876	9 N	−0.246516	17 O	−0.346139	25 H	0.165986
2 C	0.039846	10 C	0.195984	18 C	0.073556	26 H	0.013599
3 C	−0.091306	11 C	−0.107392	19 N	0.171552	27 H	0.05545
4 C	0.017922	12 C	0.167013	20 O	−0.232266	28 H	0.125148
5 C	0.178191	13 N	−0.13244	21 O	−0.251716	29 H	0.070861
6 C	0.063516	14 C	0.227604	22 H	0.032153	30 H	0.060315
7 C	0.2005	15 N	−0.268169	23 H	0.005984	31 H	0.062919
8 O	−0.121118	16 O	−0.265349	24 H	0.026436

**Table 5:** Natural population analysis (NPA) of C5NV.

	Natural	Natural Population			
Atom No	Charge	Core	Valance	Rydberg	Total
C 1	0.00881	1.9987	3.96656	0.02593	5.99119
C 2	−0.18266	1.99888	4.16533	0.01845	6.18266
C 3	−0.12894	1.9989	4.11373	0.01631	6.12894
C 4	−0.25603	1.99887	4.24005	0.01711	6.25603
C 5	0.28202	1.99865	3.69563	0.0237	5.71798
C 6	0.3726	1.99864	3.60016	0.0286	5.6274
C 7	0.19793	1.9991	3.77688	0.02608	5.80207
O 8	−0.64674	1.99975	6.63604	0.01095	8.64674
N 9	−0.5498	1.9993	5.52756	0.02294	7.5498
C 10	0.4989	1.99901	3.46991	0.03218	5.5011
C 11	−0.38383	1.99892	4.36918	0.01574	6.38383
C 12	0.10557	1.99905	3.87621	0.01918	5.89443
N 13	−0.65275	1.99926	5.64337	0.01012	7.65275
C 14	0.87323	1.99935	3.07282	0.05461	5.12677
N 15	−0.62082	1.99923	5.59939	0.02219	7.62082
O 16	−0.63298	1.99979	6.62374	0.00945	8.63298
O 17	−0.58254	1.99971	6.57263	0.0102	8.58254
C 18	−0.25739	1.99936	4.24316	0.01487	6.25739
N 19	0.52638	1.99931	4.4157	0.05861	6.47362
O 20	−0.36249	1.99979	6.34808	0.01463	8.36249
O 21	−0.39892	1.99979	6.38502	0.01411	8.39892
H 22	0.27407	0	0.72246	0.00347	0.72593
H 23	0.26429	0	0.73176	0.00395	0.73571
H 24	0.2135	0	0.78027	0.00623	0.7865
H 25	0.49757	0	0.49461	0.00782	0.50243
H 26	0.25622	0	0.741	0.00278	0.74378
H 27	0.23306	0	0.7646	0.00234	0.76694
H 28	0.43308	0	0.56151	0.00541	0.56692
H 29	0.2203	0	0.77799	0.00171	0.7797
H 30	0.1984	0	0.79841	0.00319	0.8016
H 31	0.19998	0	0.79684	0.00318	0.80002

**Fig. 8:** Mulliken population analysis (MPA) of C5NV.

**Fig. 9:** Natural population analysis (NPA) of C5NV.

### 3.16 NBO analysis

The title molecule was subjected to NBO analysis using the NBO 3.1 program employed in the Gaussian software, employing the WB97XD/cc-pVDZ level. The aforementioned work offers a viable foundation for investigating the highest electron density and electron delocalization within the molecular system orbital bonding [76]. The NBO analysis is a valuable tool for comprehending the inter- and intra-molecular interactions through the examination of exchanges between donor-acceptor orbitals within a molecule [77]. This analysis is carefully computed using second-order perturbation theory [78]. Table 6 provides a summary of the estimated donor-acceptor interactions and significant stabilization energies associated with C5NV.

**Table 6:** Natural bond orbital analysis (NBO) of C5NV.

Donar	Type	ED/e	Acceptor	Type	ED/e	E(2)^a^	E(j-i)^b^	F(i,j)^c^
C 1 - C 2	σ	1.9705	C 1 - C 6	σ*	0.03262	5.4	1.46	0.079
			C 2 - C 3	σ*	0.02235	3.71	1.5	0.067
			C 2 - H 22	σ*	0.01464	1.39	1.35	0.039
			C 3 - C 7	σ*	0.03115	4.28	1.39	0.069
			C 6 - O 8	σ*	0.01609	4.57	1.26	0.068
			N 19 - O 20	σ*	0.05552	2.36	1.36	0.051
C 1 - C 6	σ	1.97015	C 1 - C 2	σ*	0.01808	5.13	1.49	0.078
			C 1 - N 19	σ*	0.1026	0.67	1.2	0.026
			C 2 - H 22	σ*	0.01464	2.34	1.38	0.051
			C 5 - C 6	σ*	0.03925	3.6	1.44	0.064
			C 5 - O 17	σ*	0.03004	2.99	1.26	0.055
			C 6 - O 8	σ*	0.01609	1.26	1.29	0.036
			O 8 - H 25	σ*	0.02111	2.58	1.33	0.052
			N 19 - O 21	σ*	0.059	1.92	1.37	0.046
C 1 - C 6	π	1.66248	C 1 - C 6	π*	0.40563	1.27	0.4	0.021
			C 2 - C 3	π*	0.33588	37.03	0.43	0.112
			C 4 - C 5	π*	0.31677	22.98	0.42	0.088
			N 19 - O 20	π*	0.59665	25.54	0.27	0.079
C 1 - N 19	σ	1.9881	C 1 - C 2	σ*	0.01808	0.95	1.56	0.034
			C 1 - C 6	σ*	0.03262	0.89	1.56	0.033
			C 2 - C 3	σ*	0.02235	2.02	1.59	0.051
			C 5 - C 6	σ*	0.03925	2.08	1.51	0.05
C 2 - C 3	σ	1.96964	C 1 - C 2	σ*	0.01808	3.67	1.46	0.066
			C 1 - N 19	σ*	0.1026	4.89	1.18	0.069
			C 2 - H 22	σ*	0.01464	1.79	1.35	0.044
			C 3 - C 4	σ*	0.02628	4.55	1.46	0.073
			C 3 - C 7	σ*	0.03115	3.04	1.39	0.058
			C 4 - H 23	σ*	0.01647	2.74	1.34	0.054
			C 7 - N 9	σ*	0.0112	1.78	1.5	0.046
C 2 - C 3	π	1.67711	C 1 - C 6	π*	0.40563	27.13	0.38	0.092
			C 2 - C 3	π*	0.33588	0.65	0.41	0.015
			C 4 - C 5	π*	0.31677	31.53	0.4	0.1
			C 7 - N 9	π*	0.12129	26.41	0.42	0.099
C 2 - H 22	σ	1.97388	C 1 - C 2	σ*	0.01808	1	1.27	0.032
			C 1 - C 6	σ*	0.03262	5.86	1.27	0.077
			C 1 - N 19	σ*	0.1026	1.48	0.98	0.035
			C 2 - C 3	σ*	0.02235	1.57	1.3	0.04
			C 3 - C 4	σ*	0.02628	5.71	1.26	0.076
C 3 - C 4	σ	1.96509	C 2 - C 3	σ*	0.02235	4.58	1.47	0.074
			C 2 - H 22	σ*	0.01464	3.14	1.33	0.058
			C 3 - C 7	σ*	0.03115	2.87	1.37	0.056
			C 4 - C 5	σ*	0.02495	4.05	1.47	0.069
			C 4 - H 23	σ*	0.01647	1.63	1.32	0.042
			C 5 - O 17	σ*	0.03004	6.96	1.21	0.082
			C 7 - H 24	σ*	0.03432	1.75	1.31	0.043
C 3 - C 7	σ	1.97208	C 1 - C 2	σ*	0.01808	3.2	1.42	0.06
			C 2 - C 3	σ*	0.02235	3.26	1.45	0.062
			C 3 - C 4	σ*	0.02628	3.2	1.42	0.06
			C 4 - C 5	σ*	0.02495	2.73	1.45	0.056
			C 7 - N 9	σ*	0.0112	1.86	1.46	0.047
			N 9 - C 10	σ*	0.04417	4.75	1.29	0.07
C 4 - C 5	σ	1.97715	C 3 - C 4	σ*	0.02628	4.03	1.49	0.069
			C 3 - C 7	σ*	0.03115	3.69	1.42	0.065
			C 4 - H 23	σ*	0.01647	1.82	1.37	0.045
			C 5 - C 6	σ*	0.03925	5.11	1.44	0.077
			C 5 - O 17	σ*	0.03004	0.8	1.26	0.028
			C 6 - O 8	σ*	0.01609	2.78	1.29	0.053
C 4 - C 5	π	1.72248	C 1 - C 6	π*	0.40563	31.83	0.4	0.104
			C 2 - C 3	π*	0.33588	26.18	0.43	0.096
C 4 - H 23	σ	1.97327	C 2 - C 3	σ*	0.02235	5.15	1.31	0.073
			C 3 - C 4	σ*	0.02628	1.34	1.27	0.037
			C 4 - C 5	σ*	0.02495	1.42	1.31	0.038
			C 5 - C 6	σ*	0.03925	5.89	1.22	0.076
			C 5 - O 17	σ*	0.03004	0.89	1.04	0.027
C 5 - C 6	σ	1.96771	C 1 - C 6	σ*	0.03262	4.4	1.47	0.072
			C 1 - N 19	σ*	0.04417	5.7	1.18	0.075
			C 4 - C 5	σ*	0.02495	4.85	1.5	0.076
			C 4 - H 23	σ*	0.01647	3.18	1.35	0.059
			O 17 - C 18	σ*	0.00941	4.11	1.16	0.062
C 5 - O 17	σ	1.99	C 1 - C 6	σ*	0.03262	2.45	1.68	0.058
			C 3 - C 4	σ*	0.02628	1.6	1.68	0.046
			C 4 - C 5	σ*	0.02495	1.23	1.71	0.041
			C 18 - H 29	σ*	0.00682	0.82	1.55	0.032
C 6 - O 8	σ	1.99292	C 1 - C 2	σ*	0.01808	1.96	1.72	0.052
			C 1 - C 6	σ*	0.03262	1.34	1.72	0.043
			C 4 - C 5	σ*	0.02495	2.08	1.75	0.054
			C 5 - C 6	σ*	0.03925	0.91	1.67	0.035
C 7 - N 9	σ	1.98576	C 2 - C 3	σ*	0.02235	2.38	1.66	0.056
			C 3 - C 7	σ*	0.03115	1.82	1.55	0.048
			C 7 - H 24	σ*	0.03432	0.59	1.49	0.027
			N 9 - C 10	σ*	0.04417	1.83	1.49	0.047
			C 10 - C 11	σ*	0.0381	2.47	1.58	0.056
C 7 - N 9	π	1.89421	C 2 - C 3	π*	0.33588	9.6	0.49	0.065
			C 10 - N 15	π*	0.29818	1.59	1.07	0.038
			C 10 - N 15	π*	0.29818	22.14	0.48	0.097
C 7 - H 24	σ	1.98575	C 3 - C 4	σ*	0.02628	5.1	1.27	0.072
			C 10 - C 11	σ*	0.0381	0.6	1.23	0.024
			C 1 - C 6	σ*	0.03262	7.93	1.49	0.097
			C 5 - C 6	σ*	0.03925	0.8	1.44	0.03
N 9 - C 10	σ	1.9781	C 3 - C 7	σ*	0.03115	4.67	1.45	0.074
			C 7 - N 9	σ*	0.0112	1.74	1.56	0.047
			C 10 - C 11	σ*	0.0381	0.73	1.48	0.029
			C 10 - N 15	σ*	0.02821	0.89	1.53	0.033
			C 11 - C 12	σ*	0.01324	2.04	1.58	0.051
			C 14 - N 15	σ*	0.06832	3.67	1.42	0.065
C 10 - C 11	σ	1.97514	C 7 - N 9	σ*	0.0112	3.12	1.48	0.061
			N 9 - C 10	σ*	0.04417	0.94	1.31	0.032
			C 10 - N 15	σ*	0.02821	2.23	1.45	0.051
			C 11 - C 12	σ*	0.01324	2.62	1.5	0.056
			C 11 - H 26	σ*	0.01116	1.37	1.34	0.038
			C 12 - H 27	σ*	0.01386	4.6	1.31	0.07
C 10 - N 15	σ	1.98536	N 9 - C 10	σ*	0.04417	0.61	1.48	0.027
			C 10 - C 11	σ*	0.0381	2.46	1.57	0.056
			C 11 - H 26	σ*	0.01116	1.55	1.51	0.043
			C 14 - N 15	σ*	0.06832	1.29	1.52	0.04
			C 14 - O 16	σ*	0.01705	3.23	1.69	0.066
C 10 - N 15	π	1.82265	C 7 - N 9	π*	0.12129	5.43	0.48	0.046
			C 10 - N 15	π*	0.29818	0.78	0.46	0.017
			C 11 - C 12	π*	0.22505	10.4	0.47	0.063
			C 14 - O 16	π*	0.32277	39.7	0.48	0.127
C 11 - C 12	σ	1.9779	N 9 - C 10	σ*	0.04417	3.9	1.36	0.065
			C 10 - C 11	σ*	0.0381	2.79	1.45	0.057
			C 11 - H 26	σ*	0.01116	1.83	1.39	0.045
			C 12 - N 13	σ*	0.02127	1.71	1.4	0.044
			C 12 - H 27	σ*	0.01386	1.57	1.37	0.041
			N 13 - H 28	σ*	0.0163	3.66	1.34	0.063
C 11 - C 12	π	1.80352	C 10 - N 15	π*	0.29818	39.64	0.43	0.119
			C 11 - C 12	π*	0.22505	2.73	0.44	0.031
			C 14 - O 16	π*	0.32277	0.57	0.44	0.015
C 11 - H 26	σ	1.97672	N 9 - C 10	σ*	0.04417	0.62	1.14	0.024
			C 10 - C 11	σ*	0.0381	0.91	1.23	0.03
			C 10 - N 15	σ*	0.02821	5.46	1.28	0.075
			C 11 - C 12	σ*	0.01324	1.59	1.32	0.041
			C 12 - N 13	σ*	0.02127	5.69	1.17	0.073
C 12 - N 13	σ	1.98786	C 11 - C 12	σ*	0.01324	1.71	1.66	0.048
			C 11 - H 26	σ*	0.01116	2.61	1.5	0.056
			N 13 - C 14	σ*	0.10704	1.53	1.43	0.043
			N 13 - H 28	σ*	0.0163	0.92	1.46	0.033
			C 14 - O 16	σ*	0.01705	1.88	1.68	0.05
C 12 - H 27	σ	1.98077	C 10 - C 11	σ*	0.0381	4.43	1.26	0.067
			C 11 - C 12	σ*	0.01324	1.27	1.36	0.037
			N 13 - C 14	σ*	0.10704	5.66	1.12	0.073
N 13 - C 14	σ	1.98992	C 10 - N 15	σ*	0.02821	0.55	1.56	0.026
			C 12 - N 13	σ*	0.02127	2.25	1.45	0.051
			C 12 - H 27	σ*	0.01386	2.2	1.42	0.05
			N 13 - H 28	σ*	0.0163	0.52	1.4	0.024
N 13 - H 28	σ	1.98547	C 11 - C 12	σ*	0.01324	3.46	1.47	0.064
			C 14 - N 15	σ*	0.06832	3.76	1.31	0.064
			C 14 - O 16	σ*	0.01705	0.77	1.48	0.03
C 14 - N 15	σ	1.98059	N 9 - C 10	σ*	0.04417	5.44	1.4	0.078
			C 10 - N 15	σ*	0.02821	1.68	1.54	0.046
			N 13 - H 28	σ*	0.0163	2.35	1.39	0.051
			C 14 - O 16	σ*	0.01705	0.75	1.6	0.031
C 14 - O 16	σ	1.99462	C 10 - N 15	σ*	0.02821	2	1.81	0.054
			C 12 - N 13	σ*	0.02127	2.11	1.71	0.054
			C 14 - N 15	σ*	0.06832	1.04	1.7	0.038
C 14 - O 16	π	1.98838	C 10 - N 15	π*	0.29818	4.53	0.51	0.046
			C 14 - O 16	π*	0.32277	1.32	0.53	0.026
O 17 - C 18	σ	1.99178	C 5 - C 6	σ*	0.03925	3.12	1.55	0.063
C 18 - H 29	σ	1.98991	C 5 - O 17	σ*	0.03004	4.69	1.05	0.063
C 18 - H 30	σ	1.99493	C 5 - O 17	σ*	0.03004	0.58	1.05	0.022
C 18 - H 31	σ	1.99492	C 5 - O 17	σ*	0.03004	0.58	1.05	0.022
N 19 - O 20	σ	1.99475	C 1 - C 2	σ*	0.01808	0.98	1.85	0.038
			C 1 - N 19	σ*	0.04417	1.02	1.57	0.037
N 19 - O 20	π	1.98642	C 1 - C 6	π*	0.40563	3.93	0.59	0.048
			N 19 - O 20	π*	0.59665	5.85	0.46	0.055
N 19 - O 21	σ	1.99468	C 1 - C 6	σ*	0.03262	1.07	1.85	0.04
			C 1 - N 19	σ*	0.1026	0.96	1.56	0.035
LP (1)	O 8	1.97652	C 5 - C 6	σ*	0.03925	7.8	1.3	0.09
LP (2)	O 8	1.82341	C 1 - C 6	π*	0.40563	51.62	0.46	0.146
LP (1)	N 9	1.89573	C 3 - C 7	σ*	0.03115	3.01	1.01	0.05
			C 4 - H 23	σ*	0.01647	0.83	0.97	0.026
			C 7 - H 24	σ*	0.03432	14.75	0.95	0.108
			C 10 - C 11	σ*	0.0381	0.75	1.04	0.025
			C 10 - N 15	σ*	0.02821	7.92	1.09	0.085
			C 10 - N 15	σ*	0.02821	7.26	0.51	0.057
LP (1)	N 13	1.60819	C 11 - C 12	σ*	0.01324	66.86	0.41	0.155
			C 14 - O 16	σ*	0.01705	60.07	0.42	0.144
LP (1)	N 15	1.89731	C 7 - N 9	σ*	0.0112	0.53	1.1	0.022
			C 7 - H 24	σ*	0.03432	0.5	0.93	0.02
			N 9 - C 10	σ*	0.04417	7.35	0.93	0.075
			C 10 - C 11	σ*	0.0381	14.73	1.02	0.111
			N 13 - C 14	σ*	0.10704	14.06	0.88	0.099
			C 14 - O 16	σ*	0.01705	3.97	1.13	0.061
LP (1)	O 16	1.97519	N 13 - C 14	σ*	0.10704	1.79	1.21	0.042
			C 14 - N 15	σ*	0.06832	2.14	1.29	0.047
LP (1)	O 17	1.95263	C 4 - C 5	σ*	0.02495	8.21	1.35	0.095
			C 5 - C 6	σ*	0.03925	1.1	1.27	0.033
			C 18 - H 29	σ*	0.00682	2.38	1.19	0.048
			C 18 - H 30	σ*	0.01695	1.41	1.17	0.037
			C 18 - H 31	σ*	0.01679	1.38	1.17	0.036
LP (2)	O 17	1.86218	C 4 - C 5	π*	0.31677	36.33	0.49	0.125
LP (1)	O 20	1.97961	C 1 - N 19	σ*	0.1026	5.17	1.25	0.073
			N 19 - O 21	π*	0.059	2.57	1.41	0.054
LP (1)	O 21	1.97987	C 1 - N 19	σ*	0.1026	5.1	1.25	0.073
			N 19 - O 20	σ*	0.05552	2.4	1.43	0.053
LP (2)	O 21	1.89524	C 1 - C 6	π*	0.40563	0.97	1.01	0.029
			C 2 - C 3	π*	0.33588	0.73	1.05	0.025
			N 19 - O 20	π*	0.59665	23.62	0.91	0.132
LP (3)	O 21	1.45821	N 19 - O 20	σ*	0.05552	237.42	0.23	0.21
			N 19 - O 21	σ*	0.059	0.76	0.84	0.026

In this context, Ei and Ej represent the energies associated with Lewis and non-Lewis NBOs respectively [79]. F(i,j) denotes the off-diagonal component of the NBO Fock matrix, whereas qi represents the population of the donor orbital occupancy [80]. The NBO calculations conducted in this study have revealed that the target chemical exhibits two distinct forms of interactions, namely σ→ σ* and π → π* [81]. The intramolecular interaction between π(C1–C6) → π*(C2–C3) and π*(N19–O20), and π(C2–C3) → π*(C4–C5) and π*(C7–N9) exhibits significant stabilization energy, measuring at 37.03, 25.54, 31.53 and 26.41 kcal/mol, respectively. The lone pair donor (O21) in conjunction with the anti-bonding acceptor (N19–O20) exhibited the highest level of stabilization energy such as 237.42 kcal/mol.

### 3.17 Topology analysis

The nature and strength of bonding between two neighboring atoms have been characterized by examining the interaction, whether it is covalent or non-covalent. The titled compound ELF and LOL surface map are presented in Fig. 10. Denoted is the molecular graph that contains every Bond Critical Point (BCP) of the ELF [82]. The electron energy density and the negative value of the Laplacian serve as indicators of the electronic charge concentration at the Bond Critical Point (BCP) [83]. This point is characterized by the intense hydrogen bonding that occurs between atoms and is responsible for the sharing of electron pairs. Blue is employed to signify the minimum value on the scale [84]. This will cause the electron localization function (ELF) surrounding the nitrogen atom of the amino group to be distorted. The image visually signifies that the covalent regions denoted in red are responsible for generating a significant LOL value. In the ELF map, the regions surrounding carbon atoms exhibit lower values, suggesting the presence of delocalized electrons. Conversely, the regions surrounding hydrogen atoms display relatively higher values, showing the presence of localized electrons involved in bonding and non-bonding interactions [85]. Therefore, a notable ELF or LOL value is observed in the contested region, indicating a distinct electron localization caused by a covalent bond, a lone pair of electrons, or a nuclear shell. This observation suggests a modification that took place between the C–N atoms.

**Fig. 10:** ELF and LOL surface map of C5NV.

### 3.18 NCI analysis

The RDG is employed as a method to investigate the many non-covalent interactions present inside molecules. Fig. 11 illustrates the distinct zones of interaction between the titled compound. There exist three distinct domains of interaction [86]. The regions that are shown by the color green correspond to the van der Waals interactions. The red hue is indicative of repulsive interactions, mostly concentrated at the cyclic level, which can be attributed to the steric effect [87]. These interactions are predicated upon the characteristics of electron density. The presence of hydrogen bonding can be inferred from the blue patches [88]. In general, van der Waals (VDW) interactions have relatively low electron densities, whereas the regions associated with hydrogen bonding and steric effects demonstrate higher densities.

**Fig. 11:** RDG surface map of C5NV.

### 3.19 Molecular docking

In the present study, a docking analysis was conducted using metal phosphates from Danio rerio. The proteins from the Protein Data Bank (PDB) with the accession code 2XNF were chosen as the targets for the docking process [89]. The docking with the active sites of the CDP-glycerol glycerophosphotransferase inhibitor was performed using Auto-dock software [90]. The docking parameters of the amino acid residue moieties involved in interacting with the receptors are documented in Table 7, while the 2D interaction graphs are depicted in Fig. 12. Table 8 presents the binding energies [91]. The amino acid two GLN53 establishes a typical C–H bond with the O atom and N atom, with a distance of 2.39 A° and 2.38 A°. On the other hand, ARG48 makes another conventional hydrogen bond with the hydrogen atoms, respectively, exhibiting lengths of 2.0 A°. The compound carbon-hydrogen bond has one H-donor hydrogen bond with the hydrogen, located at distances of 2.76 A°, respectively [92]. Additionally, a pi-sigma interaction is observed at a distance of 3.52 A° [93]. The residue ARG51 exhibits an Amide-Pi Stacked contact with oxygen and nitrogen atoms, whereas ARG51 forms a hydrophobic pi-alkyl connection with the center at distances of 3.80 A°, respectively. The ARG48, CYS86, and VAL88 establish three hydrophobic alkyl interactions with ring centers, denoted at distances of 3.65, 4.19, and 4.68 (Å), respectively [94]. The computational analysis of molecular docking indicates that the chemical being studied demonstrates a highly favorable binding energy of −7.92 kcal/mol.

**Table 7:** Protein-ligand interaction amino acid residues of C5NV with 2XNF protein.

Distance	Category	Type	From	From-Chem	To	To-Chem
2.395	Hydrogen Bond	Conventional Hydrogen Bond	A:GLN53:HE21	H-Donor	:UNK0:O	H-Acceptor
2.38693	Hydrogen Bond	Conventional Hydrogen Bond	A:GLN53:HE21:B	H-Donor	:UNK0:N	H-Acceptor
2.20446	Hydrogen Bond	Conventional Hydrogen Bond	:UNK0:H	H-Donor	A:ARG48:O	H-Acceptor
2.76795	Hydrogen Bond	Carbon Hydrogen Bond	:UNK0:C	H-Donor	A:CYS86:O	H-Acceptor
3.52983	Hydrophobic	Pi-Sigma	A:GLN53:CG:B	C–H	:UNK0	Pi-Orbitals
4.62705	Hydrophobic	Amide-Pi Stacked	A:ARG51:C,O; VAL52:N	Amide	:UNK0	Pi-Orbitals
3.65349	Hydrophobic	Alkyl	:UNK0:C	Alkyl	A:ARG48	Alkyl
4.19265	Hydrophobic	Alkyl	:UNK0:C	Alkyl	A:CYS86	Alkyl
4.68252	Hydrophobic	Alkyl	:UNK0:C	Alkyl	A:VAL88	Alkyl
3.80762	Hydrophobic	Pi-Alkyl	:UNK0	Pi-Orbitals	A:ARG51	Alkyl

**Fig. 12:** Protein-ligand interaction sites (2D and 3D) of C5NV with 2XNF protein.

**Table 8:** Protein-ligand interaction energies of C5NV with 2XNF protein.

Rank	Run	Binding Energy	Cluster RMSD	Reference RMSD
1	28	−7.92	0	38.59
1	29	−7.88	0.65	38.71
1	12	−7.67	0.4	38.63
1	48	−7.54	1.22	38.67
1	14	−7.49	1.28	38.54
1	18	−7.35	1.35	38.44
1	4	−7.17	1.2	39.21
2	19	−6.64	0	43.56
2	24	−5.77	1.61	44
3	7	−6.47	0	41.77
3	36	−6.36	1.41	42.28
3	17	−6.17	1.67	42.76
3	47	−5.99	1.56	42.07
3	31	−5.98	1.38	42.48
4	37	−6.44	0	27.04
4	45	−6.31	0.68	27.23
4	22	−5.97	1.46	26.51
4	1	−5.95	1.77	27.57
4	46	−5.92	0.6	26.97
4	44	−5.86	0.73	27.36
4	49	−5.83	0.86	27.68
4	2	−5.82	2	27.75
4	5	−5.38	1.82	27.25
5	35	−5.87	0	35.49
6	20	−5.86	0	42.87
6	8	−5.55	1.71	42.4
7	33	−5.86	0	43.58
7	26	−5.84	1.39	44.87
7	6	−5.81	0.39	43.75
7	40	−5.59	1.25	43.5
7	13	−5.54	1.58	44.34
8	42	−5.81	0	42.94
8	39	−5.51	1.42	43.08
8	32	−5.38	1.18	43.08
9	10	−5.79	0	36.37
10	25	−5.77	0	37.21
10	3	−5.5	1.51	37.67
11	11	−5.7	0	37.11
12	15	−5.65	0	26.84
13	23	−5.61	0	48
14	9	−5.61	0	41.51
15	21	−5.57	0	31.64
16	16	−5.55	0	43.06
17	38	−5.51	0	32.79
17	27	−5.38	1.82	32.37
18	34	−5.4	0	15.73
19	41	−5.37	0	43.78
20	43	−5.36	0	37.14
21	30	−5.26	0	30.36
22	50	−5.06	0	28.91

## 4 Conclusion

An experimental and computational study was investigated on a new class of C5NV synthesized from cytosine. C5NV exhibits van der Waals interactions in both its monomeric and dimeric states. The regions of high chemical significance and the depletion region of the titled compound can be elucidated by employing the electron localization function in conjunction with the gas phase. The computed UV–Vis results exhibit excitation energies and absorption maxima. The band gap energies at all solvents have the same values, which are 2.73 eV. These findings suggest that the compound shares similarities with a drug substance. The MEP study identified the presence of electrophilic regions. This observation suggests that the titled compound possesses bioactive properties. The analysis focuses on the donor-acceptor interactions within the monomer molecule. Specifically, the stabilization of the transition bond π(C1–C6) is examined, which has an occupancy of 1.66248. Additionally, the antibonding π*(C2–C3) is considered, with an occupancy of 0.33588. The energy associated with this interaction is calculated to be 37.03 kcal/mol. The molecular docking binding energy value is determined to be −7.92 kcal/mol.

## Data availability statement

Data will be made available on the request.

## CRediT authorship contribution statement

**N. Elangovan:** Writing – review & editing, Writing – original draft, Validation, Software, Resources, Project administration, Methodology, Investigation, Formal analysis, Data curation, Conceptualization. **Natarajan Arumugam:** Writing – original draft, Supervision, Software, Funding acquisition, Formal analysis, Data curation, Conceptualization. **Abdulrahman I. Almansour:** Visualization, Validation, Project administration, Methodology, Investigation. **Shanty Mathew:** Validation, Investigation, Formal analysis, Data curation. **Sinouvassane Djearamane:** Visualization, Validation, Methodology, Investigation, Formal analysis. **Ling Shing Wong:** Visualization, Validation, Supervision, Project administration, Methodology, Investigation. **Saminathan Kayarohanam:** Validation, Supervision, Software, Resources.

## Declaration of competing interest

The authors declare the following financial interests/personal relationships which may be considered as potential competing interests:Natarajan Arumugam reports financial support was provided by 10.13039/501100002383King Saud University. Natarajan Arumugam reports a relationship with King Saud University that includes:. If there are other authors, they declare that they have no known competing financial interests or personal relationships that could have appeared to influence the work reported in this paper.
